# Doxorubicin nanobubble for combining ultrasonography and targeted chemotherapy of rabbit with VX2 liver tumor

**DOI:** 10.1007/s13277-015-4525-5

**Published:** 2016-01-06

**Authors:** Mingming Meng, Jie Gao, Chongchong Wu, Xuan Zhou, Xuefeng Zang, Xiangchun Lin, Hong Liu, Canghai Wang, Hui Su, Kuiliang Liu, Yadan Wang, Xinying Xue, Jing Wu

**Affiliations:** 1 The Department of Gastroenterology, Beijing Shijitan Hospital, Capital Medical University, 10 Tieyi Road, Yangfang District, Beijing, 100038 China; 2 The Department of Pathology, Chinese PLA General Hospital, Beijing, China; 3 The Department of Radiology, Chinese PLA General Hospital, Beijing, China; 4 The Department of Critical Care Medicine, Chinese PLA General Hospital, Beijing, China; 5 The Department of Critical Care Medicine, Beijing Shijitan Hospital, Capital Medical University, Beijing, China; 6 The Department of Special Medical Treatment, Beijing Shijitan Hospital, Capital Medical University, 10 Tieyi Road, Yangfang District, Beijing, 100038 China

**Keywords:** Ultrasound, Doxorubicin nanobubble (DOX-NB), VX2 liver tumor, Treatment

## Abstract

A new class of multifunctional nanobubble using poly(lactic-co-glycolic acid) (PLGA) has been developed as ultrasound imaging contrast agents, doxorubicin carriers, and enhancers of ultrasound-mediated drug delivery. The doxorubicin nanobubble (DOX-NB) wrapping carbon tetrafluoride gas was prepared with double emulsion method. We evaluated the enhanced ultrasonic function of the DOX-NB in vivo; its antitumor function was confirmed. The diameter of the prepared bubble was 500 nm, and the potential was −23 mV. The drug loading and encapsulation efficiency of the bubble were 78.6 and 7.4 %, respectively. Therefore, the DOX-NB greatly enhanced ultrasound imaging in vivo. Ultrasound combined with DOX-NB had significant antitumor effect. Compared with other groups, the tumor growth rate and the proliferation index were the lowest while the survival rate and apoptosis index were the highest.

## Introduction

The organ toxicity of conventional chemotherapeutic agents usually leads to relatively low level of drug concentration on target area of the body, thus limits the clinical use of chemotherapeutic drugs. In the past decade, several nanocarriers have been developed, such as liposomes, which can wrap the chemotherapeutic agents and reduce the side effects significantly. Previous studies showed that the nanodrug carriers could escape identification by reticuloendothelial system after surface modification and can keep away from the nontargeted area. Therefore, the use of nanodrug carrier cycle period has been extended [1]. Nanodrugs can pass through the endothelial gap of tumor and accumulate in tumor target area passively. Research has shown that the interval between vascular endothelial gap in a variety of tumors is between 380 and 780 nm [2, 3], and nanodrug carriers will not accumulate in normal tissue since normal tissue vascular connects more tightly with each other. In addition to higher vascular permeability, the lymphatic clearance ability of the tumor tissue is very poor, which ensures the retention of the nanoparticles in tumor tissue for a long time.

Ultrasound microbubble contrast agent is composed of gaseous core wrapping gas shell such as lipids, surfactants, and high molecular polymer. Because of the acoustic scattering properties and incidence ultrasound nonlinear function of ultrasound microbubble contrast agent, it is used to enhance ultrasound imaging [4]. Over these years, ultrasound imaging agents, such as ultrasound microbubble, has been widely used in clinical application [5–7]. In the last decade, more and more researchers demonstrated that the microbubble was used as drug carrier enhanced the delivery of drug and gene extensively [8–10]. Ultrasound microbubble contrast agent particle size must be less than 8 μm to get through the pulmonary capillaries. Ultrasound microbubble contrast agent can burst to deliver drug under certain energy ultrasound to realize the therapeutic effect. Since ultrasound microbubble contrast agent has low cost and dual role of ultrasound imaging and ultrasound-mediated therapy [11], it has become a new type of carrier in the detection and therapy of tumor. Many research teams are working on the research of ultrasound microbubble contrast agent imaging and therapeutic capabilities. However, it also has limitations, such as the cycle period of which is reduced significantly due to the dispersion of interior gas and the clearance function of body [12, 13]. In addition, the size of the microbubble is usually more than 1 μm, which limits its stay within the vascular system. As a result, it cannot reach the tumor tissue area to truly achieve tumor imaging and therapy, thus restricting its tumor target imaging and therapy application [14].

In this study, we intended to introduce a new type of nanobubbles based on poly(lactic-co-glycolic acid) (PLGA) polymer wrapping doxorubicin and carbon tetrafluoride gas that could enhance ultrasound imaging of tumor and improve ultrasound-mediated therapeutic effect. Its important feature was to integrate tumor ultrasound imaging, drug delivery, and tumor targeting. PLGA’s high stability, biodegradability, and biocompatibility in vivo enabled it a preferable choice for pharmaceutical carrier material [15–17]. Studies have confirmed that the micelles loaded with doxorubicin can be successfully released in vitro under vibration effects of certain energy ultrasound [18]. In this study, we observed the tumor ultrasound imaging effects and therapeutic properties of loading DOX-NB applied in rabbit VX2 tumor.

## Materials and methods

Double emulsion method and vacuum freeze-drying technology were used to prepare nanodoxorubicin microbubble contrast agent. One hundred milligrams of PLGA was added to 2 ml dichloromethane and stirred until completely dissolved. Then, 200 μl doxorubicin solution was added and concussion 30 s with sound and vibration analyzer until the solution became white emulsion (W/O microspheres). Of PVA solution (10 ml), 4 % was poured into the emulsion and dispersed for 5 min with the high-speed omogenizer, and then, 20 ml 2 % isopropyl alcohol solution was added to evaporate methylene chloride sufficiently. It was then washed with double-distilled water and centrifuged (5000 rpm) to collect the microspheres to obtain nanoparticles loaded with doxorubicin. Place it in a freeze drier for 48 h, and then, fill it with perfluoropropane gas to load doxorubicin nanomicrobubble contrast agent. Keep it in refrigerator under 4 °C.

### General feature detection of loaded DOX-NB

Observe morphology of nanoparticle with ordinary optical microscope and scanning electron microscope. Detect the particle size and its distribution using Malvern laser particle size analyzer. Detect Zeta potential using the surface potential cytometry.

### Detection of encapsulation efficiency and drug capacity of loaded DOX-NB

Five milligrams of loaded doxorubicin nanobubble contrast agent was dissolved into 2 ml DMSO, making nanobubble PLGA shell fully dissolved. Then, add PBS, shock 10 min, stop shaking after seeing water and oil layering. Extract the water layer, measure its absorbance value, and calculate the encapsulation efficiency and drug loading using the following formulation:

$$ \mathrm{Encapsulation}\ \mathrm{efficiency}\left(\%\right)=\mathrm{W}\mathrm{N}/\mathrm{W}\mathrm{D} \times 100\%;\ \mathrm{drug}\ \mathrm{loading}\ \left(\%\right)=\mathrm{W}\mathrm{N}/\mathrm{W}\mathrm{P} \times 100\% $$

WN is the doxorubicin content contained into the nanobubble, WD stands for the invested amount of doxorubicin, and WP is the weight of nanobubble loaded with doxorubicin.

### Assessment drug release in vitro of load DOX-NB

In order to assess the in vitro release characteristics of the loaded DOX-NB in the ultrasound field, we conducted in vitro drug release experiments using two groups, i.e., loaded DOX-NB group and ultrasonic irradiation-loaded DOX-NB group. The ultrasonic group was irradiated with ultrasonic gene transfect instrument. The parameters were set as follows: frequency 1 MHz, sound intensity 2 W/cm^2^, trigger 1 s, interval 1 s, total 2 min. Dissolve 10 mg doxorubicin nanobubble carrier powder into 5 ml of physiological saline, then put the solution into the dialysis bag with two ends closed. And then, put the dialysis bag into stoppered container filled with 100 ml of physiological saline. After ultrasonic irradiation, the container was placed in a constant temperature shaker at an oscillation speed of 100 rpm. Control group followed the same steps with the ultrasound group while free from ultrasound irradiation. Take 1 ml sample at 2, 4, 8, 12, 24, 36, 48, 60, and 72 h, respectively, and save these samples in refrigerator under 4 °C. Add 1 ml saline after taking sample every time. Then, test the doxorubicin concentration in samples at different time points by high-performance liquid chromatography, calculate the cumulative release percentage of the loaded doxorubicin nanobubble, and plot the time-concentration curve.

### Preparation of rabbit VX2 xenograft model

Take off tumor-bearing rabbits’ abdominal hairs with 3 % sodium sulfide and make the rabbit anesthesia with 2 % pentobarbital sodium. Surgical dissect VX2 rabbit liver tumor mass under sterile conditions. After rinsing several times with saline, take fresh fish-like organization and cut the tumor into 1-mm^3^ tumor mass sinking into saline solution. Open abdominal cavity of the anesthesia and abdominal hair removal rabbit in a sterile condition, expose the liver, and put the prepared tumor mass into the left lobe of the liver with ophthalmic tweezers. Stop bleeding, suture the abdominal skin layer by layer, and then intramuscular injects of 800,000 IU per animal penicillin to prevent infection for three consecutive days.

### In vivo imaging experiments of doxorubicin-contained nanobubbles

Take eight tumor-bearing rabbits and divide them into two groups randomly. The experimental group was treated with doxorubicin-contained nanobubbles, and the control group was treated with normal saline and detected by a Philips iU22 ultrasound diagnostic apparatus, the probe frequency of which was 7–10 MHz and the mechanical index was 0.1. Before ultrasound imaging, strip rabbit abdominal hair with 3 % sodium sulfide and then anesthetize the animals through intramuscular injection of 2 % sodium pentobarbital. Dissolve 100 mg of the contained DOX-NB in 1 ml saline and then inject it into rabbit by ear vein injection. At the same time, image the tumor.

### In vivo antitumor effect of doxorubicin-contained nanobubbles

In order to assess the antitumor effect of the ultrasound combined with contained doxorubicin nanobubble in vivo, we measured the tumor size of 50 tumor-bearing rabbits by two-dimensional ultrasonography scanning 15 days after VX2 carcinoma modeling. Divide the animals into five groups randomly, i.e., control group, doxorubicin group, ultrasound group, doxorubicin-loaded nanobubble group, and ultrasound combined with doxorubicin-loaded nanobubble group. Provide different treatments to groups for the first 16, 18, and 20 days, respectively. The treatment schedule was as follows: inject 2 ml of saline by ear vein to the control group, inject 2 ml of doxorubicin solution to doxorubicin group, inject 2 ml DOX-NBs to doxorubicin-loaded nanobubble group. Ultrasound combined with doxorubicin-loaded nanobubble was not only injected with 2 ml DOX-NBs but was also surface orientation irradiated VX2 tumors under two-dimensional ultrasound monitoring using ultrasound gene transfection instrument. Parameters were set as follows: frequency 1 MHz, sound intensity 2 W/cm^2^, trigger 1 s, interval 1 s, total 2 min.

Therapeutic method of ultrasound group was the same as the ultrasound combined with doxorubicin group and without injection of DOX-NB. Tumor volume (V) was calculated according to the following equation: *V* = (*L* × *S* ^2^) / 2. *L* and *S* stood for the maximum and minimum diameter of the tumor, respectively. Tumor growth curve was plotted based on the change of the tumor volume. After the observation, four rabbits in each group were sacrificed and tumor mass was stripped. The tumor mass was sliced and fixed with 4 % of paraformaldehyde. After embedded with paraffin, the expression of apoptosis and proliferation of cells in tumor tissue was detected by immunohistochemical assay and the expression of apoptosis cell was detected by terminal deoxynucleotidyl transferase dUTP nick end labeling (TUNEL) assay, and the death index and proliferation index were calculated according to the following formula. The remained rabbits continued to be observed to death. Record the survival time of each group to draw KM survival curves, thus comparing the survival ratio in each group. The study was approved by the Ethics Committee of Beijing Shijitan Hospital.

## Results and discussion

In this study, we observed that the PLGA DOX-NB could enhance the imaging of tumors under ultrasound and work as a drug carrier in ultrasound-mediated treatment. The doxorubicin was prepared with double emulsion method. Doxorubicin was introduced to the reaction medium prior to PVA. The introduced carbon tetrafluoride gas equipped the bubble with the characteristics of ultrasound imaging. After intravenous injection of DOX-NB to tumor-bearing VX2 rabbit, ultrasound gene transfect device could emit certain energy ultrasonic wave to burst the nanobubbles or accelerate drug release of the nanobubbles, thus enhancing the concentration of doxorubicin in tumors to achieve the antitumor effect. The existence of carbon tetrafluoride gas could enhance the precision of ultrasound imaging and drug release under the two-dimensional ultrasound monitoring.

We evaluated the size, potential, and surface characteristics of DOX-NB (Fig. 1). Under scanning electron microscopy, the highly dispersed nanobubbles were observed to turn into spherical bubbles. As shown in Fig. 1, the average size of nanoparticle was 500 nm detected by dynamic scattering assay. The size of the nanoparticle was the key factor of whether it could pass through the endothelial gap in liver. The size of our nanoparticle was between 380 and 780 nm, ensuring that the DOX-NB can achieve the tumor tissue for imaging and treatment through the EPR effect [19–23]. The potential determined the stability of DOX-NB. In this study, the potential of nanobubbles was −23 mV, which was detected by laser surface potential, so the nanoparticle was difficult to gather and had better stability. According to the determination by high-performance liquid chromatography, the encapsulation efficiency of the DOX-NB was 78.6 % while the efficiency of drug loading was 7.4 %. Figure 2 compared the drug release characteristic of DOX-NB with or without ultrasonic influence in order to confirm that ultrasound is helpful for the drug release. The drug release curve showed that the cumulative drug release rate of doxorubicin under ultrasonic vibration was faster than DOX-NB alone. About 80 % of doxorubicin was released in 24 h after ultrasound, while only 60 % of doxorubicin was released in DOX-NB group. Meanwhile, we calculated the time for 50 % of doxorubicin to release. Under the ultrasound, it took 8 h for 50 % doxorubicin to release while it needed 12 h without ultrasound. Within the first 12 h, we found that the burst release happened in both ultrasonic group and control group. The drug release rate of the two groups was 70 and 50 %, respectively. From 12 to 72 h, the drug release rate was stable. At 72 h, the drug release rate of ultrasound rate reached 90 % while the control group was only 70 %. The results confirmed that ultrasound had controlled release effect for DOX-NB, and doxorubicin nanoparticle could deliver drug targeting at tumor under the monitoring of ultrasound. Some studies also confirmed that the underlying mechanism of ultrasound triggering release of drug from doxorubicin nanoparticle was that ultrasound could accelerate the degradation of PLGA [24].

**Fig. 1:** **a** Light microscopy images of DOX-NB, **b** scanning electron microscopy (SEM) images of DOX-NB, **c** size distribution of DOX-NB by dynamic light scattering (DLS) measurement, and **d** potential distribution of DOX-NB by DLS measurement

**Fig. 2:** The release curve of DOX-NB between ultrasound and no ultrasound in vitro

In the in vivo VX2 liver cancer imaging process, compared with saline, DOX-NB could enhance the ultrasonic imaging significantly in tumor area. After the ear vein injection of DOX-NB, the nanobubbles could quickly attain the tumor area and reach the peak after 17 s (Fig. 3). This result confirmed that DOX-NB could be used to enhance ultrasound imaging in clinic and release drug to the targeted tissue under the two-dimensional ultrasound monitoring.

**Fig. 3:** The time intensity curve of DOX-NB in the VX2 liver tumor

Fifteen days after planting VX2 tumor cells into rabbits, tumor was successfully inoculated in the left lobe of the liver and the diameters of all tumors were more than 10 mm. According to the tumor growth curve (Fig. 4), the tumor growth rate was the fastest in control group and the ultrasound group while the rate was the slowest in the ultrasound combined with DOX-NB group. Compared with the control group, the inhibitory rate of ultrasound combined with DOX-NB group is 76.7 %, doxorubicin-loaded nanobubble group is 57.4 %, doxorubicin group is 45.3 %, and ultrasound group is 15 %. After anticancer treatment, tumor volume in ultrasound combined with DOX-NB group was significantly smaller than the other groups, while the tumor volume inhibition rate was the highest among three groups. The tumor growth in both doxorubicin group and ultrasound combined with DOX-NB group was suppressed. However, the inhibitory rate in ultrasound combined with DOX-NB group was higher than the nanobubble group. These findings confirmed that the tumor therapeutic effect of doxorubicin nanobubble was poor without the effect of ultrasound. The possible reason may be the low drug release rate in tumor area, thus leading to low level of doxorubicin concentration in tumor area. Both doxorubicin group and doxorubicin nanobubble group had suppressive effect to tumor, but the inhibitory effect of doxorubicin nanobubble group was better than doxorubicin group. Based on this result, we could infer that doxorubicin had intensive toxic side effects to the body after intravenous injection, which results in poor therapeutic effect. However, loading the doxorubicin into PLGA could reduce its toxicity to the body significantly, thus improving the tumor therapeutic effect to a certain extent. Immunohistochemistry results showed that proliferation cells were observed in all groups and apoptosis and proliferation index in ultrasound combined with DOX-NB group were lower than other groups (Fig. 5). The proliferation index was significantly different between each group (Fig. 6). TUNEL showed that there were apoptosis cells in tumor area in all groups and the apoptosis index in ultrasound combined nanobubble group was the highest (Fig. 7). The apoptotic index was significantly different as well (Fig. 8). The survival curves of each group showed that the survival rate in ultrasound combined nanobubble group was obviously higher than other groups (Fig. 9). Since the apoptosis index negatively correlated to the degree of tumor growth and the proliferation index positively correlated to the degree of tumor growth, the above results confirmed that the ultrasound combined with DOX-NB could significantly improve the anticancer therapeutic effect.

**Fig. 4:** Tumor growth curve of liver tumor

**Fig. 5:** The different expression of PCNA in each group using immunohistochemical staining. **a** Control group, **b** US group, **c** DOX group, **d** DOX-NB, and **e** DOX-NB + US group

**Fig. 6:** The proliferation index of each group VX2 liver tumor cell

**Fig. 7:** Cell apoptosis in each group VX2 liver tumor by TUNEL. **a** Control group, **b** US group, **c** DOX group, **d** DOX-NB, and **e** DOX-NB + US group

**Fig. 8:** Apoptotic index of VX2 liver tumor cells in each group

**Fig. 9:** KM survival curves of VX2 liver tumor cells in each group

In summary, we fabricated DOX-NB based on PLGA composites successfully. Doxorubicin nanobubble can be used as ultrasound contrast agent to enhance tissue imaging. Meanwhile, its application can suppress VX2 tumor growth significantly in vivo. Therefore, DOX-NB has great potential in tumor therapy mediated by two-dimensional ultrasound and provides a new insight for tumor imaging and therapy.

## References

[1] Bekeredjian R, Chen S, Frenkel PA, Grayburn PA, Shohet RV (2003). Ultrasound-targeted microbubble destruction can repeatedly direct highly specific plasmid expression to the heart. Circulation.

[2] Burns PN, Wilson SR, Simpson DH (2000). Pulse inversion imaging of liver blood flow: improved method for characterizing focal masses with microbubble contrast. Investig Radiol.

[3] Campbell RB (2006). Tumor physiology and delivery of nanopharmaceuticals. Anticancer Agents in Med Chem.

[4] Eisenbrey JR, Burstein OM, Kambhampati R, Forsberg F, Liu JB, Wheatley MA (2010). Development and optimization of a doxorubicin loaded poly(lactic acid) contrast agent for ultrasound directed drug delivery. J Control Release.

[5] El-Sherif DM, Lathia JD, Le NT, Wheatley MA (2004). Ultrasound degradation of novel polymer contrast agents. J Biomed Mater Res A.

[6] Greish K (2007). Enhanced permeability and retention of macromolecular drugs in solid tumors: a royal gate for targeted anticancer nanomedicines. J Drug Target.

[7] Hobbs SK, Monsky WL, Yuan F, Roberts WG, Griffith L, Torchilin VP (1998). Regulation of transport pathways in tumor vessels: role of tumor type and microenvironment. Proc Natl Acad Sci U S A.

[8] Hoff L (1999). Acoustic properties of ultrasonic contrast agents. Ultrasonics.

[9] Iyer AK, Khaled G, Fang J, Maeda H (2006). Exploiting the enhanced permeability and retention effect for tumor targeting. Drug Discov Today.

[10] Jain RA (2000). The manufacturing techniques of various drug loaded biodegradable poly(lactide-co-glycolide) (PLGA) devices. Biomaterials.

[11] Kabalnov A, Bradley J, Flaim S, Klein D, Pelura T, Peters B (1998). Dissolution of multicomponent microbubbles in the bloodstream: 2. Experiment. Ultrasound Med Biol.

[12] Kabalnov A, Klein D, Pelura T, Schutt E, Weers J (1998). Dissolution of multicomponent microbubbles in the bloodstream: 1. Theory. Ultrasound Med Biol.

[13] Klibanov AL (2006). Microbubble contrast agents: targeted ultrasound imaging and ultrasound-assisted drug-delivery applications. Investig Radiol.

[14] Lawrie A, Brisken AF, Francis SE, Cumberland DC, Crossman DC, Newman CM (2000). Microbubble-enhanced ultrasound for vascular gene delivery. Gene Ther.

[15] Lindner JR (2004). Microbubbles in medical imaging: current applications and future directions. Nat Rev Drug Discov.

[16] Lindner JR, Song J, Xu F, Klibanov AL, Singbartl K, Ley K (2000). Noninvasive ultrasound imaging of inflammation using microbubbles targeted to activated leukocytes. Circulation.

[17] Matsumura Y, Maeda H (1986). A new concept for macromolecular therapeutics in cancer chemotherapy: mechanism of tumoritropic accumulation of proteins and the antitumor agent smancs. Cancer Res.

[18] Price RJ, Skyba DM, Kaul S, Skalak TC (1998). Delivery of colloidal particles and red blood cells to tissue through microvessel ruptures created by targeted microbubble destruction with ultrasound. Circulation.

[19] Ravi Kumar MN, Bakowsky U, Lehr CM (2004). Preparation and characterization of cationic PLGA nanospheres as DNA carriers. Biomaterials.

[20] Roberts WG, Palade GE (1997). Neovasculature induced by vascular endothelial growth factor is fenestrated. Cancer Res.

[21] Wilson K, Homan K, Emelianov S (2012). Biomedical photoacoustics beyond thermal expansion using triggered nanodroplet vaporization for contrast-enhanced imaging. Nat Commun.

[22] Fang J, Nakamura H, Maeda H (2011). The EPR effect: unique features of tumor blood vessels for drug delivery, factors involved, and limitations and augmentation of the effect[J]. Adv Drug Deliv Rev.

[23] Acharya S, Sahoo SK (2011). PLGA nanoparticles containing various anticancer agents and tumour delivery by EPR effect[J]. Adv Drug Deliv Rev.

[24] Yoo HS, Oh JE, Lee KH, Park TG (1999). Biodegradable nanoparticles containing doxorubicin-PLGA conjugate for sustained release. Pharm Res.

